This article has been retracted.

# Intra-articular injection in the knee of adipose derived stromal cells (stromal vascular fraction) and platelet rich plasma for osteoarthritis

**DOI:** 10.1186/s12967-017-1242-4

**Published:** 2017-06-19

**Authors:** Himanshu Bansal, Kristin Comella, Jerry Leon, Poonam Verma, Diwaker Agrawal, Prasad Koka, Thomas Ichim

**Affiliations:** 1 RegennMed Research and Therapeutics LLP, Chattarpur, Delhi, India; 2 US Stem Cell, Inc, Sunrise, FL USA; 3 Advance Health Institute Mayaguez, Puerto Rico, USA; 4 Mercy Medical Centre, Roseburg, OR USA; 5 Department of Virology and Immunology, Haffkine Institute, Mumbai, Maharashtra 400012 India; 6 Regenerative Medicine Institute, Tijuana, Mexico; 7 Mother Cell Spinal Injury & Stem Cell Research, Anupam Hospital, Second Floor, Kashipur Bypass Road, Rudrapur, Uttarakhand 263153 India

**Keywords:** Stromal vascular fraction (SVF), Adipose derived stromal/stem cells (ADSCs), Stem cells, Adipose tissue, Connective tissue, Osteoarthritis, Cell therapy, Platelet rich plasma (PRP)

## Abstract

**Background:**

Stromal vascular fraction (SVF) can easily be obtained from a mini-lipoaspirate procedure of fat tissue and platelet rich plasma (PRP) can be obtained from peripheral blood. We evaluated the safety and preliminary efficacy of administering SVF and PRP intra-articularly into patients with osteoarthritis grade 1 and 2.

**Methods:**

A total of ten patients underwent a local tumescent liposuction procedure to remove approximately 100 ml of fat tissue from the abdomen. SVF was isolated using an enzyme digestion and resuspended in PRP for intra-articular injection in the knee. The Western Ontario and McMaster Universities Osteoarthritis Index (WOMAC) score and six-minute walk distance (6MWD) were used to evaluate clinical effects and included measure of patient’s subjective assessment of pain, joint mobility, and physical disability. WOMAC score, 6MWD and laboratory tests were repeated at 3 and 6 months and 1, 1.5 and 2 years. XRAY and MRI were completed at 1 year.

**Results:**

The average total WOMAC score was 64 at baseline and significantly reduced to 52 at 3 months, 46 at 6 months, 42 at 1 year, 38 at 1.5 years, and 41 at 2 years. Patients walked an average of 1310 feet at baseline and demonstrated a statistically significant improvement at 3 and 6 months and 1, 1.5, and 2 years post treatment. Cartilage thickness as determined by MRI improved by at least 0.2 mm in six patients, was unchanged in two patients and decreased by at least 0.2 mm in two patients.

**Conclusions:**

Overall, all of the patients were pleased with the treatment results. They reported a reduction in pain levels, especially after 3 months. More importantly, the procedure demonstrated a strong safety profile with no severe adverse events or complications reported.

*Trial registration* NCT03089762; Name of registry: http://www.clinicaltrials.gov

## Background

Osteoarthritis (OA) is a degenerative disease characterized by the slow progressive destruction of articular cartilage accompanied by changes to synovium and sub chondral bone, degeneration of ligaments and menisci and hypertrophy of the joint capsule [1, 2]. The pathogenesis is usually characterized by severe inflammation, recruitment of inflammatory cells, pro inflammatory cytokine production and activation of proteinase that results in extracellular matrix (ECM) degradation and ultimately apoptotic cell death of differentiated chondrocytes. OA is influenced by genes, environment (e.g. aging and obesity) and local trauma (e.g. consequences of joint injury/joint laxity or mal-alignment). These factors and more may contribute to the pathological process involved in the degeneration of the knee [3, 4].

Typical treatments include weight reduction, rest, exercise, non-steroidal anti-inflammatory drugs (NSAIDS), intracellular glucocorticoid injections, visco supplements, physical therapy and bracing. These modes of treatments are usually palliative and merely provide symptomatic relief from pain, failing to prevent cartilage damage and subsequent destruction of other joint tissues [5–7].

Surgical methods of repair include the transplantation of osteochondral grafts, microfracture, and autologous chondrocyte implantation. All of these techniques are limited to the repair of focal lesions. According to controlled clinical trials, arthroscopic surgery, autologous chondrocyte implantation or microfracture have limited long term effect on the treatment of OA [7, 8]. The challenge for researchers to develop disease-modifying OA treatments is, therefore, of paramount importance. Adult mesenchymal stem cells (MSCs) have emerged as a candidate cell type with great potential in regenerative medicine [9]. MSCs are being investigated as a regenerative biologic agent because of their ability to differentiate into multiple tissue types and to self-renew [10, 11].

The paracrine activity of MSCs is thought to be one of the major means by which these cells mediate anti-inflammatory, anti-apoptotic, anti-fibrotic, angiogenic, mitogenic and wound healing properties. The complex interplay of the biological mediators secreted by MSCs has been shown to be important in regulating regeneration of a variety of damaged or diseased organs and tissues of the body. It has also been shown that the pre-curser to the MSC is the pericyte which are the cells present on the microvessels and capillaries throughout the body. These cells become “activated” when an injury is recognized and detach to become medicinal MSCs. An immune-modulatory effect is initiated where other cells are called to help with the healing process while other secreted molecules will establish a regenerative microenvironment by setting up a trophic field [12].

MSCs are also capable of suppressing an immune response by suppressing the maturation of dendritic cells. MSCs may also restrain the T, B, and NK cell function in inflammation. MSCs are involved in cross talk between the immune cells and as a result may present a novel approach for the treatment of various diseases [13].

The stromal vascular fraction (SVF) can be obtained from fat tissue and contains a variety of different types of cells including adipose-derived stem cells. Adipose-derived stem cells or ADSCs are multi-potential in that they have the ability to differentiate into a variety of different types of tissue including but not limited to bone, cartilage, muscle, ligament, tendon and fat [14]. These cells have also been shown to express a variety of different growth factors and signaling molecules (cytokines), which recruit other stem cells to facilitate repair and healing of the affected tissue. ADSCs are very angiogenic in nature and can promote the growth of new blood vessels. ADSCs might play a role in the local inflammatory process in the joint.

The SVF might play a role in the local inflammatory process in the joint. Studies have shown that SVF exerts anti-inflammatory effects on both chondrocytes and synoviocytes and that the cells are not dependent on adipose tissue sources or donors. SVF has been shown to exhibit immunosuppressive properties and release anti-inflammatory molecules like IL-10, IL-1, receptor antagonist (IL-1ra), indoleamine 2,3-dioxygenase, transforming growth factor (TGF) β and prostaglandin E2. The cells in SVF seem to be able to sense and respond to the local environment in OA knees [15, 16]. A stromal vascular fraction can easily be isolated from fat tissue in approximately 30–90 min in a clinic setting using a mini-lipoaspirate technique. The SVF contains a mixture of cells including ADSCs and growth factors and has been depleted of the adipocyte (fat cell) population. It has been shown that cells isolated from the SVF contain an abundance of CD34+ cells [15, 17]. SVF can be used in a point of care setting for a variety of indications and is currently being used in thousands of clinics world-wide with varying degrees of success being reported. Adipose tissue is quickly becoming the preferred source for point of care treatments in clinic due to the high number of MSCs that can be obtained and the low number of leukocytes as compared to bone marrow. In addition, adipose tissue has a significantly higher amount of pericytes which are the precursors to MSCs [18–20].

Recent studies evaluating ADSCs as a potential for articular cartilage regeneration have shown the potential of the cells to develop into chondrogenic lineage [21]. Clinical studies have reported improvements in function and pain of the knee joint as well as increased cartilage thickness with a strong safety profile [22–27].

Adipose tissue has many advantages in comparison to bone marrow. Adipose can be easily obtained by standard liposuction under local anesthesia. Adipose tissue contains approximately 500–2500 times more mesenchymal stem cells compared to the same volume of bone marrow [20]. In addition, the number of stem cells available in the bone marrow decreases with age and the pool in adipose tissue is quite stable during life. Compared with bone marrow-derived cells, adipose tissue-derived cells are more genetically stable, have higher proliferative and differentiation capacity, have lower senescence ratio, and have longer telomere length [28, 29].

In one clinical study reporting on 18 patients (between the ages of 18 and 75), SVF from subcutaneous abdominal fat was injected intra-articularly into idiopathic osteoarthritic knees. The high dose injections (1.0 × 10^8^) were associated with an improvement in pain, stiffness and function as measured by the WOMAC score with a mean reduction of 39% over a 6 month period. MRI examination found regeneration of articular cartilage in the medial femoral and tibial condyles as well as in the lateral femoral and tibial condyles and increased cartilage volume in the medial femoral and tibial condyles at 6 months. Arthroscopy before and 6 months after SVF injection demonstrated findings consistent with clinical and radiological outcomes showing the regeneration of articular cartilage with a thick, glossy white matrix and smooth surface well integrated with the sub chondral bone [24].

Another clinical study reported on 18 patients (6 men and 12 women) injected with SVF from the infrapatellar fat pad with a mean of 1.8 million cells (range 0.3 × 10^6^–2.7 × 10^6^) along with approximately 3.0 ml of platelet rich plasma with a mean of 1.28 × 10^6^ platelets/ml. OA index scores decreased significantly (p < 0.001) from 49.9 points preoperatively to 30.3 points at the final follow up (range 24–26 months). Lysholm score improved significantly from a mean preoperative value of 40.1 points to 73.4 points, and similarly VAS scores decreased from 4.8 preoperatively to 2.0 at last follow up. In addition, notable changes were detected in cartilage MRI scores which improved from 28.3 points to 21.7 points. This study suggested that intra-articular injection of SVF from infrapatellar fat pad is effective for reducing pain and promoting new tissue growth [22]. The same group had reported on an earlier study with similar results [30].

In one large trial (n = 1128), SVF was utilized in patients with grade 2–4 degenerative osteoarthritis (OA). The trial demonstrated a strong safety profile with no severe adverse events or systemic infection. In addition, no patients developed cancer as a result of SVF therapy. A majority of the patients demonstrated gradual improvement 3–12 months after the treatment. At least 75% score improvement was noticed in 63% of patients and at least 50% Score improvement was documented in 91% of patients after 12 months. The authors concluded that SVF therapy is a novel and promising treatment approach for patients with OA [26].

Adult stem cells require various growth factors to maintain their growth and engraftment. Recent studies have discussed the use of platelet rich plasma (PRP) as a rich source of growth factors. Platelets contain key growth factors such as platelet derived growth factor (PDGF), transforming growth factor (TGF), fibroblast growth factor (FGF), and various interleukins (IL) which may contribute to the functionality of the stem cells [31]. Platelet released growth factors regulate endogenous hyaluronic acid (HA) synthesis, thereby protecting the cartilage and lubricating the join [11]. It also enhances the secretion of HA and induces hepatocyte growth factor production by synovial fibroblasts isolated from arthritic patients. This study considers the intra-articular injection of SVF from fat and the safety and efficacy for the treatment of OA in combination with PRP.

## Methods

The criteria for selection were patients age 50 or older who present with symptomatic primary osteoarthritis of the knee [1], defined by daily pain for the previous 3 months, analgesics usage at least once a week, less than 30 min of morning stiffness and a WOMAC score of ≤75 in the target knee. The radiographic eligibility criteria included Brandt Radiographic Grading Scale of Osteoarthritis grade 1 and 2. The exclusion criteria were evidence of secondary knee osteoarthritis, severe osteoarthritis (joint space width—JSW <2 mm), prior intra articular injections within the previous 1 year prior to inclusion and patients with clinically significant systemic disease.

The Western Ontario and McMaster Universities Osteoarthritis Index (WOMAC) is a widely used measure of patient’s subjective assessment of pain, joint mobility and physical disability. It evaluates three dimensions, namely pain, stiffness and physical function with 5, 2, and 17 questions respectively. Total maximum score is 96 and minimum is 0. Each subscale is summated to a maximum score of 20, 8 and 68 respectively [32].

The six-minute walking distance (6MWD) was carried out by marking off a 50 m distance in an interior hallway and asking subjects to walk as far as they can and as quickly as they can over 6 min. The total distance was measured and recorded [33].

Antero-posterior radiographs of the knee joints were obtained with patients in a weight bearing position, joint fully extended, standing at 1 m from the X-Ray source, using previously published guidelines. Width was measured at the narrowest point of the joint space width (minimal JSW). This progression was defined by a JSW loss of more than 0.50 mm during the study, as previously reported [34].

MRI was completed with 1.5 T standard protocols of each individual joint in coronal sagittal and transverse plane. Maximum thickness of cartilage at posterior/meniscal and patellar level measured at mid sagittal thru medial condyle was taken into account. The medial femoral cartilage of the affected knee was selected for measurement. Three regions of the medial femoral condyle were identified at the anterior patella femoral, meniscal and posterior condyle level. The point having maximum thickness in the sagittal section passing thru the middle was identified for measurement.

Etoricoxib with a dose limited 90 mg BD after meals was advised to patients for unbearable pain. If the pain was still uncomfortable then they were advised to take codeine in a dose of 30 mg as needed and report the next day.

Tolerability and safety assessments included any symptoms and signs reported by the patient and also laboratory based hematological and biochemical assays. Synovial fluid was analyzed using microscopic examination at baseline and 2 years post procedure for atypical cell counts. Adverse events were categorized as isolated, intermittent or continuous depending on interference with the subject’s daily activities as mild, moderate or severe. Possible causal relationship with the supplement in terms of Definite/Possible/Probable/Non Assessable/None were assigned. The study was approved by institutional committee for stem cell research and therapy. All the patients were well informed and gave written consent to participate in the study.

### Isolation of stromal vascular fraction cells from adipose tissue

From each patient, approximately 100 ml fat was collected from the abdomen using a 3 mm aspiration cannula with prior administration of tumescent solution and placed into sterile disposable 250 ml conical centrifuge tubes. The adipose tissue was washed twice in phosphate buffered saline (PBS) and digested using collagenase at 37 °C for 30 min with agitation at 5-min intervals. The suspension was then divided into four 50 ml centrifuge tubes and centrifuged at 500×*g* for 5 min to collect the SVF as a pellet. The pellet was washed twice with normal saline to remove any residual enzyme, and resuspended in PBS. The SVF suspension was filtered through a 100 μm cell strainer and centrifuged at 500×*g* for 5 min. The supernatant was discarded. The pellet was resuspended in normal saline and filtered through a 40 µm cell strainer. Samples were taken to determine the cell quantity, viability, and to culture and characterize the stem cells.

### Culture of the cells

The cells were washed thoroughly with DPBS/Gentamycin thoroughly twice. These were centrifuged at 1500 rpm for 10 min. Supernatant was discarded. The pellet was re-suspended in complete DMEM medium (Sigma) and plated in a T25 flask and incubated at 37 °C under 5% CO_2_. Media was changed every 3–4 days until the cells achieved 90% confluency. The cells were characterized through morphological evaluation and flow cytometry analysis.

### Morphological studies

The cells were cultured in six well plates up to 70% confluency in complete DMEM media and pictures were taken at different time intervals by an inverted microscope at 20× magnification.

### Flow cytometry studies

For flow cytometry, the cells were cultured in six well plates in complete DMEM media to 80% confluency. These were harvested using mild trypsin EDTA and washed with PBS. The cells were incubated with fluorescently labeled antibodies CD90, CD34, CD73, CD45, CD105 and HLA-DR. The cells were processed for flow cytometry analysis using BD FACS Calibur.

### Platelet rich plasma preparation

Platelet rich plasma was derived from the peripheral blood of the same donor as the adipose tissue. Briefly, 20 ml of peripheral blood was collected into BD yellow top vacuum tubes (ACD Solution A) and centrifuged at 800×*g* for 10 min. The plasma fraction was collected and centrifuged at 1000×*g* for 5 min to obtain a platelet pellet. Most of the plasma was then removed, leaving 3 ml plasma to resuspend the platelets.

### Statistical analysis

Formal power calculations were not performed. Two tailed statistical analyses were performed and confidence intervals are presented with 95% degree of confidence. All statistical tests used a significance level of α ≤0.05.

### Treatments

A total of ten patients over the age of 50 with idiopathic osteoarthritis of the knee were enrolled in the study. SVF cells were resuspended in 5 ml of saline and combined with 3 ml of PRP. A single injection of SVF and PRP was administered intra-articularly. At the baseline, patients were assessed for vital signs, laboratory tests, WOMAC score, 6MWD, radiological images of joint space width, and MRI measurement of articular cartilage thickness. Clinical status of all patients was closely monitored at baseline, at the time of SVF treatment, 1 week, 1, 3, 6 months, and 1, 1.5 and 2 years after the SVF treatment. WOMAC score, 6 MWD and laboratory tests were repeated at 3 and 6 months and 1, 1.5 and 2 years. XRAY and MRI were completed at 1 year. Clinical evaluation included medical history, physical examination, assessment of joint pain, number of analgesic drugs taken, joint stiffness and extent of joint movement, as well as any side effects possibly associated with SVF cell therapy.

## Results

A total of ten patients were treated with mean age of 58.4, height of 158.2 cm and weight of 72.6 kg. Six patients were male and four were female. Seven patients had one knee treated and three had both knees injected. Fat harvested yielded an average nucleated SVF mean cell concentration of 1 × 10^6^/ml of adipose tissue and viability of 87.4%. The morphology of the cultured cells appeared to be like typical fibroblastic mesenchymal stem cells adhered to the plastic surface (Fig. 1a). Few clumps of the cells were observed. The flow Cytometry data show more than 98% positive expression of CD105, CD90 and CD73 and negative expression of CD45, CD34 and HLA DR (Fig. 1b).

**Fig. 1:** **a** Morphology of the fat derived MSC. **b** Flow cytometry analysis of MSC using BD FACS calibur

Significant changes in the WOMAC scores were noted in both the subsets and the total after 2 years as compared to the baseline. A correlation between pain severity and disability was demonstrated by the WOMAC subscales. The WOMAC scale allows a detailed analysis of pain because patients score the pain severity while performing specific activities. Patients had a decreased functional ability most likely due to severe pain at baseline readings. The average total WOMAC score (Fig. 2a) was 64 at the baseline and significantly reduced to 52 at 3 months (p < 0.01), 46 at 6 months (p < 0.01), 42 at 1 year (p < 0.01), 38 at 1.5 years (p < 0.01), and 41 at 2 years (p < 0.01).

**Fig. 2:** **a** Total WOMAC score. **b** WOMAC pain score. **c** WOMAC stiffness score. **d** WOMAC physical function score

WOMAC pain score during walking, using stairs, in bed, sitting or lying and standing were also recorded. Patients demonstrated a significant reduction in pain (Fig. 2b) from 14 at baseline to 12 at 3 months (p < 0.01), 11 at 6 months (p < 0.01), 9 at 1 year (p < 0.01), 8 at 1.5 years (p < 0.01), and 9 at 2 years (p < 0.01) post therapy. Stiffness score (Fig. 2c) which includes 17 parameters, showed reduction from 6 at baseline to 5 at 3 months and 6 months (p < 0.01), and 4 at 1, 1.5 and 2 years (p < 0.01). Physical function score (Fig. 2d) of 50 from the baseline reduced to 44 at 3 months (p < 0.01), 38 at 6 months (p < 0.01), 32 at 1 year (p < 0.01), 30 at 1.5 years (p < 0.01) and 31 at 2 years (p < 0.01).

Figure 3 shows the results of the 6MWD. Patients walked an average of 1310 feet at baseline and demonstrated a statistically significant improvement (p < 0.01) at 3 and 6 months and 1, 1.5, and 2 years post treatment. In addition, the requirement of pain medication post injection reduced from twice a week at baseline to once a week in 3 patients at 3 months, 5 patients at 6 months, 7 patients at 1 year, 8 patients at 1.5 years and 5 patients at 2 years.

**Fig. 3:** Six minute walk distance (6MWD)

MRI evaluation demonstrated that cartilage thickness improved by at least 0.2 mm in six patients. Thickness remained unchanged in two patients at 1 year, which indicated chondro-protective and anti-inflammatory disease stabilization effect. However, in two patients it decreased by 0.2 mm. At 2 years post injection, one patient received a follow up MRI which showed that the increased cartilage volume was maintained (Fig. 4). Figures 5, 6, 7, 8 show MRIs at baseline and 1 year post treatment.

**Fig. 4:** MRI **a** baseline, **b** 2 years post injection. Improvement of 0.2 mm at posterior condyle/meniscus sites

**Fig. 5:** MRI **a** baseline, **b** 12 months post injection. Improvement of 0.2 mm at meniscus and patellar

**Fig. 6:** MRI **a** baseline, **b** 12 months post injection. Improvement of 0.2 mm at posterior and meniscus. No changes noted at patella/femoral level

**Fig. 7:** MRI **a** baseline, **b** 12 months post injection. Improvement of 0.2 mm at posterior level. No changes noted in anterior level or meniscus

**Fig. 8:** MRI **a** baseline, **b** 12 months post injection. Improvement at all levels

Overall, all of patients were pleased with the treatment results. They reported that their pain levels gradually reduced, especially after 3 months. More importantly, the procedure demonstrated a strong safety profile with no severe adverse events or complications reported. One patient complained of pain and swelling due to reactive synovitis which responded with complete resolution with conservative treatment.

### Safety evaluation

Two years post procedure, synovial fluid examination showed no atypical cells (Table 1). However, the analysis suggested that treatment helped to restore synovial fluid properties, restore synovial metabolism and reduce cartilage pathology. Eight patients demonstrated a reduction in atypical cells. Average cell counts were 1226 cells/μl at baseline and reduced to 845 cells/μl at 2 years. The hematological and biochemical parameters recorded before and after 2 years of the treatment also did not show any abnormalities (Table 2).

**Table 1:** Number of atypical cells/μl

Baseline	At 2 year follow up
1440	490
680	460
860	560
1200	800
1600	880
1780	1260
460	480
1060	440
1380	1260
1800	1820
Average	
1226	845

**Table 2:** Hematological and biochemical parameters

Parameter	Baseline	2 years
RBC count, 10^6^/μl	4–4.6	4.2–4.6
Hemoglobin, g/dl	12–14.2	11.6–14.4
PCV heamtocrit, %	38–40	36–42
Platelet count, 1000/μl	260–340	250–380
White blood cell count, 1000/μl	6.4–8.4	6.6–8.6
WBC differential count		
Neutrophils, %	56–70	60–70
Eosinophils, %	2–6	1–6
Lymphocytes, %	30–38	32–36
Monocytes	2–3	1–3
Basophils	0	0
CRP	<1	<1
ESR	8–14	10–14
SGPT, IU/l	28–32	28–38
SGOT, IU/l	16–20	18–20
Serum creatinine, mg/dl	0.5–0.9	0.6–0.9
Glucose (F)	90–110	86–108

## Discussion

Osteoarthritis is a chronic progressive degenerative disease associated with cartilage loss and degeneration. Current treatments are limited and advanced disease relies on total joint replacement. Total joint replacement may be associated with serious and life threatening complications including increased risk of infection, thrombo-embolism, myocardial infarction, stroke, and even death post-surgery. In addition, the life span of the prosthesis is limited [34].

This preliminary clinical study showed that SVF cells freshly isolated from adipose tissue, combined with PRP and administered intra-articularly, demonstrate healing potential in patients with degenerative OA. This is consistent with previously published results from both preclinical and clinical studies. Patients demonstrated significant improvements in their degenerative OA leading to a better quality of life. These improvements included a clinically significant reduction in pain.

Pain functional status of the knee was improved 12 months post injection in all patients and this improvement was maintained at the 2 year time point. Some patients showed improvements as early as 3 and 6 months after the injection of SVF and PRP. This confirms the mechanism of action of regenerative medicine to be a cascade of events that occur over time. These events include an immuno-modulatory effect that can lead to tissue remodeling. The anti-inflammatory and pain reduction effects may be attributed to the soluble growth factors secreted from the SVF or ADSCs [32]. Growth factors from ADSCs may be continuously produced after injection of these cells into the joint creating a cascade of events that lead to healing. It is unclear at this point whether the cells injected actually differentiate into new cartilage or the cells injected stimulate native tissue to heal by creating a paracrine effect. Native cells may be called to the area to help remodel the damaged tissue leading to an increase in cartilage volume [11].

The autologous SVF and PRP injections also significantly reduced the requirement of pain medication in 8 out of 10 patients. These medications are often associated with undesired side effects and although it may mask the pain, it does not help the underlying disease. In addition, clinical improvement corresponded well with improvement on MRI imaging. We were able to demonstrate safety with no serious side effects reported during the 2 year follow-up. One patient experienced local pain and swelling at the lipo-aspiration site, but those symptoms were short lasting and were well controlled with common analgesics. Only one patient developed synovitis in the joint which resolved with conservative treatment.

Freshly isolated cells may represent a safe and efficacious way to manage patients with osteoarthritis. An immediate autologous transplantation can prevent complications related to the reduced quality of the transplanted cells such as pre-aging (telomere shortening), reduced viability, or dedifferentiation/reprogramming that is associated with in vitro-cultivation [35]. In addition, the risk for infection is reduced by decreasing the ex vivo time period. Although in this study cells isolated from SVF were also evaluated by culture and characterization to further establish existence of MSCs in the fraction, cells isolated from SVF expressed characteristics distinctive for MSC identification such as plastic adherence with typical fibroblast like morphology and positive MSC markers by flow cytometry. Overall the entire treatment is a relatively simple procedure which is inexpensive and can be completed in clinic on an outpatient basis. Numerous studies are currently in progress to clarify some of the questions that still remain unanswered regarding the long-term durability of these procedures and possible modifications to achieve better results. Here we present preliminary data suggesting safety and long term efficacy of a cost effective outpatient procedure of administration of SVF and PRP in the knee.

This study lacks a placebo control due to very small sample size. The relationship of age, sex, weight and the severity of OA could not be clearly ascertained. In addition, MRI evaluation should have been more extensive with three-dimensional magnetic resonance observation of cartilage repair tissue (MOCART) or other scaling methods to quantify the regeneration in cartilage following the treatment. Further it is not clear if the regenerated cartilage is fibro cartilage or hyaline as arthroscopic biopsy was not possible in any of subjects. The extensive pathologic changes in OA were identified as “joint failure” not only in articular cartilage but also in the changes of synovial membrane. Changes in subchondral bone and joint capsules were not investigated.

## Conclusions

SVF combined with PRP has a great potential as a therapeutic agent in regenerative medicine especially in orthopedic conditions. The high numbers of MSCs in SVF make it a suitable source for cellular medicine. Preliminary studies suggest that it is a safe and effective method for treating osteoarthritis. Both qualitative and quantitative measurements showed statistically significant improvements during the follow up period of 2 years. Additional studies with larger patient numbers and control subjects are needed to confirm the above results. Another limitation of this study is the combined effects of two modalities is unclear. Future studies with randomized groups considering each therapeutic agent separately and combined against a control are warranted. This clinical study of a combined intra-articular injection of SVF and PRP into the knee suggests a promising minimally invasive therapy for OA patients.

## Abbreviations

SVF: stromal vascular fraction
PRP: platelet rich plasma
ADSCs: adipose derived stem/stromal cells
MSC: mesenchymal stem cell
WOMAC: Western Ontario and McMaster Universities Osteoarthritis Index
6MWD: six-minute walk distance
MOCART: magnetic resonance observation of cartilage repair tissue
SAE: severe adverse event
OA: osteoarthritis
